The article "miR-182-5p Serves as an Oncogene in Lung Adenocarcinoma through Binding to STARD13" was retracted in 2023. Reasons: signs of a paper mill; suspected computer-generated content; unreliable results or conclusions; lack of ethics approval or compliance.

# miR-182-5p Serves as an Oncogene in Lung Adenocarcinoma through Binding to STARD13

**DOI:** 10.1155/2021/7074343

**Published:** 2021-07-22

**Authors:** Xuhui Wu, Wei Wang, Gongzhi Wu, CongXiong Peng, Jichun Liu

**Affiliations:** ^1^Department of Cardiothoracic Surgery, The First Affiliated Hospital of Nanchang University, Nanchang, Jiangxi Province, China 330006; ^2^Department of Emergency and Critical Care Medicine, The Second Affiliated Hospital of Nanchang University, Nanchang, Jiangxi Province, China 330006; ^3^Department of Cardiothoracic Surgery, The Sixth Affiliated Hospital of Wenzhou Medical University, Lishui, Zhejiang Province, China 323000

## Abstract

Lung cancer as one of the commonest invasive malignancies is featured by high morbidity and mortality, wherein lung adenocarcinoma (LUAD) is the most prevalent subtype. Accumulating evidence exhibited that microRNAs are involved in LUAD occurrence and progression. In this study, miR-182-5p was observed to increase in both LUAD tissue and cell lines. Overexpression of miR-182-5p could prominently facilitate cell proliferation, migration, and invasion in LUAD. Through bioinformatics analysis, STARD13 was theorized as the target gene of miR-182-5p, which was lowly expressed in LUAD. Further molecular experiments manifested that miR-182-5p bound to the 3′-untranslated region of STARD13, and there was an inverse correlation between STARD13 and miR-182-5p in LUAD. Rescue experiments demonstrated that silencing STARD13 conspicuously restored the inhibitory effect of decreased miR-182-5p on cell proliferation, migration, and invasion in LUAD. Together, our findings revealed novel roles of the miR-182-5p/STARD13 axis in LUAD progression.

## 1. Introduction

Lung adenocarcinoma (LUAD) as the most prevalent histological subtype of lung cancer is responsible for 40% of all lung cancer cases. It has high metastasis and invasive potential, with a poor 5-year survival [1]. Deepgoing study of the pathology of LUAD is of primary importance in current scientific research. Seeking out novel targets for molecular therapy through basic research can provide fresh diagnostic and prognostic strategies for LUAD, which can militate early diagnosis of LUAD patients and improve therapeutic efficacies.

Numerous cellular biological functions such as cell differentiation, development, progression, and apoptosis are determined by a class of small noncoding RNAs, namely, microRNAs (miRNAs) [2, 3]. Through inversely regulating gene expression at the posttranscriptional level, miRNAs can repress gene translation and lead to direct degradation of mRNAs [4]. miR-182-5p as a neotype cancer-related miRNA is extensively reported to play a regulatory role in various kinds of tumors. Cao et al. [5] observed that increased miR-182-5p in hepatocellular carcinoma tissue and cells facilitates cancer cell proliferation, migration, and invasion through FOXO3a suppression. Li et al. [6] found that miR-182-5p is upregulated in oral squamous cell carcinoma (OSCC) cells and clinical samples, as well as functions as an oncogene in OSCC via hindering CAMK2N1 expression. miR-182-5p is identified as an oncogene in ovarian cancer [7], breast cancer and [8], melanoma [9], whereas it exerts an inhibitory role in renal cell carcinoma [10, 11] and bladder cancer [12]. Regarding different roles of miR-182-5p in different tumors, it may be due to the heterogeneity of different tumors. In non-small-cell lung cancer (NSCLC), miR-182 acts an oncogenic role and fosters cell proliferation by directly targeting FBXW7 and FBXW11, indicating that miR-182 may be a fresh diagnostic and prognostic biomarker of NSCLC [13]. However, there are few detailed investigations of the regulatory mechanism of miR-182-5p and its role in LUAD.

The article "miR-182-5p Serves as an Oncogene in Lung Adenocarcinoma through Binding to STARD13" was retracted in 2023. Reasons: signs of a paper mill; suspected computer-generated content; unreliable results or conclusions; lack of ethics approval or compliance.

In this study, we identified StAR-related lipid transfer protein 13 (STARD13), the target gene that had the strongest negative correlation with miR-182-5p, as the research object by bioinformatics analysis. STARD13, namely, DLC2, located on chromosome 13q12.3, is the GTPase-activating protein for Rho, and it has been proven to be a tumor repressor [14]. For instance, STARD13 is downregulated in prostate cancer, and its overexpression hinders proliferation of cancer cells [15]. It is also considered a tumor repressor in hepatocellular carcinoma [16]. However, no relevant reports focused on STARD13 in LUAD.

This study deeply investigated the expression and molecular mechanism of miR-182-5p and STARD13 in LUAD, and our results may lay a theoretical basis for the discovery of therapeutic targets underlying LUAD.

## 2. Materials and Methods

### 2.1. Bioinformatics Analysis

Expression profiles of mature miRNAs (normal: *n* = 45; tumor: *n* = 513), as well as mRNA sequencing data (normal: *n* = 58; tumor: *n* = 519), were downloaded from The Cancer Genome Atlas (TCGA) database. Differential analysis was conducted by using R package “edgeR,” with the normal samples as control. With ∣logFC | >1.5 and adj.*p*value < 0.05 as thresholds for selecting differentially expressed miRNAs (DEmiRNAs), the miRNA of interest was determined. Then, the downstream target genes of the target miRNA were predicted through TargetScan, mirDIP, miRDB, miRWalk, and starBase databases. Meanwhile, based on gene expression in TCGA-LUAD, downregulated differentially expressed RNAs (DEmRNAs) in LUAD were intersected with the predicted results to screen out the target mRNA, thereby determining the miRNA-mRNA regulatory pair.

The article "miR-182-5p Serves as an Oncogene in Lung Adenocarcinoma through Binding to STARD13" was retracted in 2023. Reasons: signs of a paper mill; suspected computer-generated content; unreliable results or conclusions; lack of ethics approval or compliance.

### 2.2. Cell Culture

Human LUAD cell lines A549 (BNCC341254), Calu-3 (BNCC338514), PC-9 (BNCC340767), and PAa (BNCC341415) and human bronchial epithelial cell line BEAS-2B (BNCC338205) were all purchased from BeNa Culture Collection (BNCC). A549 and PAa cells were prepared in Roswell Park Memorial Institute-1640 (RPMI-1640) medium. Calu-3 cells were cultured in Minimum Essential Medium-Earle's Balanced Salts Solution (MEM-EBSS). PC-9 and BEAS-2B cells were cultivated in Dulbecco's Modified Eagle Medium-high glucose (DMEM-H) medium. The mediums used in this study all contained 10% fetal bovine serum (FBS) and were supplemented with 100 U/ml streptomycin (Gibco; Thermo Fisher Scientific, Inc.) and 100 U/ml penicillin (Gibco; Thermo Fisher Scientific, Inc.). Cells were cultured in an incubator at 37°C, with 5% CO_2_.

### 2.3. Cell Transfection

miR-182-5p mimic and miR-182-5p inhibitor and their corresponding negative controls were all accessed from Sangon Biotech (Shanghai, China). When cells grew to 50% confluence, the synthetic sequence miR-182-5p mimic/mimic NC was transiently transfected into LUAD cell A549, and miR-182-5p inhibitor/inhibitor NC was transiently transfected into PC-9 cells as per the instructions of Lipofectamine 2000 (Invitrogen, Carlsbad, CA, USA). The medium was replaced 4-6 h after transfection. The lentivirus expression vector pLVX-IRES-neo (Clontech, USA) was utilized to construct si-STARD13 and si-NC vectors, and then, the vectors were transfected into corresponding cells.

### 2.4. RNA Isolation and Real-Time Quantitative Polymerase Chain Reaction (qRT-PCR)

Total RNA was extracted from cells by using TRIzol reagent (Invitrogen, Thermo Fisher Scientific, Inc., Waltham, MA, USA) following the manufacturer's protocol. It was quantified with a NanoDrop 2000 spectrophotometer (Thermo Fisher Scientific, Inc., Waltham, MA, USA). The SuperScript II first-strand cDNA synthesis kit (Thermo Fisher Scientific, Inc., Waltham, MA, USA) was implemented for reverse transcription. qRT-PCR was carried out on SYBR Green PCR Mix (Applied Biosystems, Foster City, CA, USA) and ABI Prism 7900 Detection System (Thermo Fisher Scientific, Inc., Waltham, MA, USA). Primer sequences used in the assay as detailed in Table 1 were purchased from Sangon Biotech (Shanghai, China). U6 and *β*-actin were used as endogenous references for miR-182-5p and STARD13, respectively. The results were presented with 2^-*ΔΔ*Ct^ value. The experiment was performed in triplicate.

### 2.5. Western Blot

Total proteins were isolated through radioimmunoprecipitation assay (RIPA) (Beyotime, Shanghai, China), and the concentration of which was measured by bicinchoninic acid (BCA) protein assay kit (Pierce Biotechnology, Rockford, IL, USA). The isolated proteins were separated on 10% sodium dodecyl sulfate polyacrylamide gel electrophoresis (SDS-PAGE) and then transferred onto polyvinylidene fluoride (PVDF) membrane (Millipore, Billerica, MA, USA). Then, 5% skim milk was recommended for membrane blockage. The membrane was incubated with specific primary antibodies at 4°C overnight and rinsed three times with phosphate-buffered saline+Tween-20 (PBST) (Beyotime, Shanghai, China), followed by incubating with horseradish peroxidase- (HRP-) labeled secondary antibody for 2 h. Finally, the immunoreactive bands were visualized through the enhanced chemiluminescence (ECL) method (Thermo Fisher, Waltham, MA, USA). Antibody information is as follows: primary antibodies rabbit anti-STARD13 (ab126489, 1 : 200, Abcam, Cambridge, UK) and *β*-actin (ab115777, 1 : 2500, Abcam, Cambridge, UK); secondary antibody goat anti-rabbit IgG H&L (HRP) (Ab205718, 1 : 2000, Abcam, Cambridge, UK).

The article "miR-182-5p Serves as an Oncogene in Lung Adenocarcinoma through Binding to STARD13" was retracted in 2023. Reasons: signs of a paper mill; suspected computer-generated content; unreliable results or conclusions; lack of ethics approval or compliance.

### 2.6. Dual-Luciferase Reporter Gene Assay

The targeting relationship between miR-182-5p and STARD13 was verified via dual-luciferase reporter gene assay. The mutant (MUT) 3′-untranslated region (3′-UTR) sequence of STARD13 was constructed by point mutation method. Then, the wild-type (WT) or MUT 3′-UTR sequences were inserted into the downstream of pmiRGLO (Promega, WI, USA) luciferase vector, and thus, the luciferase reporter plasmids STARD13-WT and STARD13-MUT were constructed. LUAD cell lines A549 and PC-9 were seeded into 24-well plates and cultured for 24 h at 37°C. Later, miR-182-5p mimic/mimic NC and STARD13-WT/MUT were cotransfected into A549 cells, while miR-182-5p inhibitor/inhibitor NC and STARD13-WT/MUT were cotransfected into PC-9 cells. Renilla luciferase expression vector pRL-TK (TaKaRa, Dalian, China) was used as an internal reference. After 48 h of transfection, the relative luciferase activity was assessed with a dual-luciferase detection kit (Promega, Madison, WI, USA).

### 2.7. Cell Counting Kit-8 (CCK-8) Assay

The transfected cells were seeded in 96-well plates at a density of 2 × 10^3^ cells/well. After 0, 24, 48, 72, and 96 h, 10 *μ*l CCK-8 solution (Dojindo, Kumamoto, Japan) was added to each well for another 2 h of cell culture. The optical density (OD) value at 450 nm was detected by a microplate reader (Bio-Rad, Hercules, CA, USA).

### 2.8. Wound Healing Assay

Cells were inoculated to 6-well plates (2.5 × 10^5^ cells/well). After cells grew to complete confluence, a 200 *μ*l pipette tip was implemented to softly scrape on the cell monolayer to make artificial wounds. The scraped cells were washed off with PBS. The wound healing was observed and photographed after 0 and 24 h.

The article "miR-182-5p Serves as an Oncogene in Lung Adenocarcinoma through Binding to STARD13" was retracted in 2023. Reasons: signs of a paper mill; suspected computer-generated content; unreliable results or conclusions; lack of ethics approval or compliance.

### 2.9. Cell Invasion Assay

Transwell chambers (BD Biosciences) precoated with Matrigel® were recommended to evaluate cell invasion. Approximately 2 × 10^4^ cells were inoculated to the upper chamber coated with Matrigel (Corning, NY) and cultured in serum-free culture medium, while the lower chamber was supplemented with 10% FBS. Twenty-four hours later, cells that passed through the Matrigel membrane were fixed and then stained with crystal violet. The number of invading cells was counted in 5-random fields under the microscope.

### 2.10. Statistical Analysis

Data management and analysis were conducted on SPSS 21.0 statistical software. Measurement data were presented as mean ± standard deviation, and the comparison between two groups adopted *t*-test, while multigroup comparison was carried out by one-way analysis of variance. *p* < 0.05 meant that the differences were statistically significant.

## 3. Results

### 3.1. miR-182-5p Is Notably Upregulated in LUAD Tissue and Cells

From mature miRNA expression data of LUAD in TCGA database, it was theorized that miR-182-5p was remarkably upregulated in LUAD tissue (Figure 1(a)), and the difference was significant compared with normal tissue. To investigate the underlying role of miR-182-5p in the malignant progression of LUAD, qRT-PCR was conducted to assess miR-182-5p expression in various LUAD cell lines. As illustrated in Figure 1(b), compared with human bronchial epithelial cell line (BEAS-2B), there was an increased miR-182-5p expression in human LUAD cell lines (A549, Calu-3, PC-9, and PAa). A549 and PC-9 cells were chosen for subsequent assays.

### 3.2. miR-182-5p Hastens Cell Proliferation, Migration, and Invasion of LUAD

To further study the biological function of miR-182-5p in LUAD cells, miR-182-5p mimic/mimic NC was transfected into the A549 cell line while miR-182-5p inhibitor/inhibitor NC was transfected into the PC-9 cell line, thereby achieving miR-183-5p overexpression/silencing artificially. As presented in Figure 2(a), each group had favorable transfection efficacy of miR-182-5p and could be used for follow-up assays. The result of CCK-8 assay manifested that miR-182-5p overexpression facilitated the proliferation of A549 cells, whereas silencing miR-182-5p decreased the proliferation of PC-9 cells (Figure 2(b)). The result of wound healing assay exhibited that the upregulation of miR-182-5p fostered LUAD cell migration while silencing miR-182-5p dramatically hampered cell migration (Figure 2(c)). Transwell assay also pointed out that the invasive ability of A549 cells in the miR-128-5p mimic group was notably enhanced in the miR-128-5p mimic group, while that of PC-9 cells in the miR-128-5p inhibitor group was markedly downregulated (Figure 2(d)). Hence, it could be concluded that miR-182-5p affected cell proliferation, migration, and invasion of LUAD, which played a pivotal role in LUAD progression.

The article "miR-182-5p Serves as an Oncogene in Lung Adenocarcinoma through Binding to STARD13" was retracted in 2023. Reasons: signs of a paper mill; suspected computer-generated content; unreliable results or conclusions; lack of ethics approval or compliance.

### 3.3. STARD13 Is Lowly Expressed in LUAD and Is a Downstream Target of miR-182-5p

To further investigate the downstream regulatory mechanism of miR-182-5p, the downstream target genes of miR-182-5p were predicted through 5 public databases (TargetScan, miRDB, starBase, mirDIP, and miRWalk). First, differential analysis was performed on genes in TCGA-LUAD dataset, and 533 downregulated DEmRNAs were intersected with predicted mRNAs to obtain 4 target genes (Figure 3(a)), among which STARD13 had the strongest inverse correlation with miR-182-5p (Figure 3(b)) and was prominently lowly expressed in cancer tissue (Figure 3(c)). Therefore, STARD13 was selected as the potential regulatory target of miR-182-5p. Later, qRT-PCR and western blot assays were carried out to detect STARD13 mRNA and protein levels in different LUAD cell lines. As presented in Figures 3(d) and 3(e), compared with the human bronchial epithelial cell line (BEAS-2B), STARD13 mRNA and protein levels were notably decreased in human LUAD cell lines (A549, Calu-3, PC-9, and PAa). Through analysis in the TargetScan database, it was found that 3′-UTR of STARD13 mRNA had complementary region with miR-182-5p (Figure 3(f)). Subsequently, dual-luciferase reporter gene assay was utilized for validation of the binding of miR-182-5p and STARD13. The result manifested that miR-182-5p mimic resulted in marked downregulation of luciferase activity of cells in the STARD13-WT mRNA 3′-UTR group, while it had no significant impact on luciferase activity of the STARD13-MUT group. Besides, miR-182-5p inhibitor led to increased luciferase activity of cells in the STARD13-WT group whereas no obvious change was observed in the STARD13-MUT group (Figure 3(g)), indicating that miR-182-5p may downregulate STARD13 gene expression through binding to STARD13 3′-UTR. Moreover, western blot also presented that miR-182-5p mimic decreased STARD13 expression in A549 cells, while miR-182-5p inhibitor increased STARD13 expression in PC-9 cells (Figure 3(h)). These results demonstrated that miR-182-5p could downregulate STARD13 expression.

### 3.4. miR-182-5p Affects Cell Proliferation, Migration, and Invasion through Modulating STARD13

To investigate whether miR-182-5p hastens the malignant progression of PC-9 cells via targeting STARD13, si-STARD13 and miR-182-5p inhibitor were cotransfected into PC-9 cells. First, qRT-PCR was conducted to assess miR-182-5p and STARD13 mRNA expression. Meanwhile, western blot was performed to measure STARD13 protein expression. The results pointed out that when miR-182-5p was inhibited, there was an increase in STARD13 mRNA and protein levels (Figures 4(a) and 4(b)). Next, a trail of experiments was conducted to validate our predictions. CCK-8 assay illustrated that compared with the miR-182-5p inhibitor+si-NC group, si-STARD13 and miR-182-5p inhibitor cotransfection could restore the proliferative activity of PC-9 cells (Figure 4(c)). Wound healing assay manifested that silencing miR-182-5p led to a decrease in LUAD cell migration, while simultaneously silencing miR-182-5p and STARD13 rescued cell migratory ability (Figure 4(d)). Transwell invasion assay revealed that compared with the inhibitor NC+si-NC group, cell invasive ability was hindered by silencing miR-182-5p while it was rescued by silencing miR-182-5p and STARD13 at the same time (Figure 4(e)). Together, these findings demonstrated that miR-182-5p modulated the proliferation, migration, and invasion of PC-9 cells via targeting STARD13.

The article "miR-182-5p Serves as an Oncogene in Lung Adenocarcinoma through Binding to STARD13" was retracted in 2023. Reasons: signs of a paper mill; suspected computer-generated content; unreliable results or conclusions; lack of ethics approval or compliance.

## 4. Discussion

miRNAs are confirmed to regulate gene expression related to tumor development, proliferation, apoptosis, and stress response [17–20], with aberrant expression in numerous human cancers. In this study, through data analysis of TCGA-LUAD, miR-182-5p was found to be prominently differentially expressed in LUAD, and its downstream inversely regulated gene STARD13 was unearthed. Most importantly, this study focused on the targeting relationship between miR-182-5p and STARD13, thereby improving regulatory mechanism of miR-182-5p in LUAD at the molecular level.

Several studies reported the role of miR-182-5p in varying cancer progression [21, 22]. For instance, miR-182-5p facilitates cell viability, mitosis, migration, and invasion in human gastric cancer through RAB27A downregulation [23]. In the present study, miR-182-5p expression was assessed and found to be conspicuously upregulated in LUAD cells. A study [8] reported that upregulated miR-182-5p serves as an oncogene in breast cancer that hastens cancer cell proliferation and migration. Besides, miR-182-5p is also upregulated in NSCLC tumor samples, which fosters the malignant progression of cancer cells by AGER suppression, and its high expression is associated with dismal prognosis of NSCLC patients [24]. In this study, miR-182-5p overexpression facilitated the proliferation, migration, and invasion of A549 cells, while silencing miR-182-5p hindered malignant progression of PC-9 cells.

The article "miR-182-5p Serves as an Oncogene in Lung Adenocarcinoma through Binding to STARD13" was retracted in 2023. Reasons: signs of a paper mill; suspected computer-generated content; unreliable results or conclusions; lack of ethics approval or compliance.

Afterwards, the downstream target mRNAs of miR-182-5p were predicted. Since miR-182-5p had the highest inverse correlation with STARD13, it was speculated that miR-182-5p may affect the malignant progression of LUAD through modulating STARD13. STARD13 or START-GAP2 is also known as DLC2 gene. Ching et al. [25] found, for the first time, that STARD13 is lowly expressed in hepatocellular carcinoma. STARD13 has a C-terminal START domain and an N-terminal SAM domain, and it holds a GAP domain for Rho GTPases between the two domains [25–27]. STARD13 as a kind of tumor-suppressive protein inhibits breast cancer cell growth, exerts an antimetastasis effect, and represses RhoA activity [28]. STARD13 modulates the Raf-1-ERK1/2-p70S6K signaling pathway in liver cancer to hinder cancer cell growth and migration [29]. In this study, compared with human bronchial epithelial cell line BEAS-2B, STARD13 was lowly expressed in LUAD cell lines. Dual-luciferase reporter gene assay verified that miR-182-5p could directly target 3′-UTR of STARD13. In addition, STARD13 expression was remarkably downregulated with overexpressing miR-182-5p, which was the opposite when silencing miR-182-5p. Cellular functional assays also authenticated that silencing miR-182-5p hindered cell proliferative, migrative, and invasive abilities, whereas this effect was restored in the miR-182-5p inhibitor+si-STARD13 group.

Overall, miR-182-5p played a pivotal role in the malignant progression of LUAD cells, and its expression affected the metastatic activity of LUAD cells. STARD13 as a tumor suppresser gene was the target protein of miR-182-5p. In a word, miR-182-5p modulated the malignant progression through targeting STARD13. These findings suggested that STARD13 may be a potential therapeutic target of LUAD. In the following investigations, we will verify whether STARD13 modulates the malignant progression of LUAD through signal pathways such as STARD13-RhoA-ROCK, thereby laying the groundwork for the treatment of LUAD.

## Figures and Tables

**Figure 1:** miR-182-5p is highly expressed in LUAD tissue and cells. (a) Box plot of miR-182-5p expression in normal (*n* = 45) and tumor (*n* = 513) tissue samples from TCGA-LUAD. (b) miR-182-5p expression in human bronchial epithelial cell line (BEAS-2B) and human LUAD cell lines (A549, Calu-3, PC-9, and PAa). ^∗^*p* < 0.05; ^∗∗∗∗^*p* < 0.0001.

**Figure 2:** miR-182-5p hastens cell proliferation, migration, and invasion of LUAD. (a) miR-182-5p expression in A549 and PC-9 cell lines detected via qRT-PCR after transfection. (b) CCK-8 assay was used to assess the proliferative ability of cells in different transfection groups (mimic NC, miR-182-5p mimic, inhibitor NC, and miR-182-5p inhibitor). (c) Wound healing assay was performed to detect the migratory ability of cells in different transfection groups. (d) Invasion assay was conducted to measure the invasive ability of cells in different transfection groups (×100). ^∗^*p* < 0.05.

The article "miR-182-5p Serves as an Oncogene in Lung Adenocarcinoma through Binding to STARD13" was retracted in 2023. Reasons: signs of a paper mill; suspected computer-generated content; unreliable results or conclusions; lack of ethics approval or compliance.

**Figure 3:** STARD13 is lowly expressed in LUAD and is a downstream target of miR-182-5p. (a) The intersection of target genes of miR-182-5p predicted by 5 databases and downregulated DEmRNAs. (b) Heatmap of correlation of miR-182-5p and the predicted genes. (c) Box plot of STARD13 expression level in normal (*n* = 58) and tumor (*n* = 519) groups. (d, e) STARD13 mRNA and protein expression levels in the human bronchial epithelial cell line (BEAS-2B) and human LUAD cell lines (A549, Calu-3, PC-9, and PAa). (f) The binding sites of miR-182-5p and STARD13. (g) The binding of miR-182-5p and STARD13 verified by dual-luciferase reporter gene assay. (h) Western blot measured the effect of overexpression/silencing of miR-182-5p on STARD13 expression. ^∗^*p* < 0.05; ^∗∗∗∗^*p* < 0.0001.

**Figure 4:** miR-182-5p affects cell proliferation, migration, and invasion through modulating STARD13. (a) qRT-PCR assessed miR-182-5p and STARD13 mRNA expression of PC-9 cells in each transfection group (inhibitor NC+si-NC, miR-182-5p inhibitor+si-NC, and miR-182-5p inhibitor+si-STARD13). (b) Western blot measured STARD13 protein expression in each transfection group. (c) CCK-8 detected cell proliferation of LUAD in each transfection group. (d) Wound healing assay assessed cell migration of LUAD in each transfection group. (e) Invasion assay measured cell invasion of LUAD in each transfection group (×100). ^∗^*p* < 0.05.

**Table 1:** Primer sequences in qRT-PCR.

Gene	Primer sequence (5′⟶3′)
miR-182-5p	F: ACACTCCAGCTGGGTTTGGCAATGGTAGAACT
	R: TGGTGTCGTGGAGTCG
U6	F: CTCGCTTCGGCAGCACA
	R: AACGCTTCACGAATTTGCGT
STARD13	F: AGCCCCTGCCTCAAAGTATT
	R: AGCCCCTGCCTCAAAGTATT
*β*-Actin	F: ATGAAGATCCTGACCGAGCGT
	R: AACGCAGCTCAGTAACAGTCCG

## Data Availability

The data used to support the findings of this study are included within the article. The data and materials in the current study are available from the corresponding author on reasonable request.

## References

[1] Vucic E. A., Pikor L. A., Enfield K. S. S. (2014). Smoking status impacts microRNA mediated prognosis and lung adenocarcinoma biology. *BMC Cancer*.

[2] Arunkumar G., Deva Magendhra Rao A., Manikandan M. (2018). Dysregulation of miR-200 family microRNAs and epithelial-mesenchymal transition markers in oral squamous cell carcinoma. *Oncology Letters*.

[3] Lee R. C., Feinbaum R. L., Ambros V. (1993). The *C. elegans* heterochronic gene _lin-4_ encodes small RNAs with antisense complementarity to _lin-14_. *Cell*.

The article "miR-182-5p Serves as an Oncogene in Lung Adenocarcinoma through Binding to STARD13" was retracted in 2023. Reasons: signs of a paper mill; suspected computer-generated content; unreliable results or conclusions; lack of ethics approval or compliance.

[4] O'Shea J. J., Holland S. M., Staudt L. M. (2013). JAKs and STATs in immunity, immunodeficiency, and cancer. *The New England Journal of Medicine*.

[5] Cao M. Q., You A. B., Zhu X. D. (2018). Correction to: miR-182-5p promotes hepatocellular carcinoma progression by repressing FOXO3a. *Journal of Hematology & Oncology*.

[6] Li N., Nan C. C., Zhong X. Y. (2018). miR-182-5p promotes growth in oral squamous cell carcinoma by inhibiting CAMK2N1. *Cellular Physiology and Biochemistry*.

[7] Xu X., Ayub B., Liu Z. (2014). Anti-miR182 reduces ovarian cancer burden, invasion, and metastasis: an in vivo study in orthotopic xenografts of nude mice. *Molecular Cancer Therapeutics*.

[8] Li P., Sheng C., Huang L. (2014). MiR-183/-96/-182 cluster is up-regulated in most breast cancers and increases cell proliferation and migration. *Breast Cancer Research*.

[9] Segura M. F., Hanniford D., Menendez S. (2009). Aberrant miR-182 expression promotes melanoma metastasis by repressing FOXO3 and microphthalmia-associated transcription factor. *Proceedings of the National Academy of Sciences of the United States of America*.

[10] Xu X., Wu J., Li S. (2014). Downregulation of microRNA-182-5p contributes to renal cell carcinoma proliferation via activating the AKT/FOXO3a signaling pathway. *Molecular Cancer*.

[11] Wang X., Li H., Cui L., Feng J., Fan Q. (2016). MicroRNA-182 suppresses clear cell renal cell carcinoma migration and invasion by targeting IGF1R. *Neoplasma*.

[12] Wang F., Wu D., Xu Z. (2019). miR-182-5p affects human bladder cancer cell proliferation, migration and invasion through regulating Cofilin 1. *Cancer cell international*.

[13] Chang H., Liu Y. H., Wang L. L. (2018). MiR-182 promotes cell proliferation by suppressing FBXW7 and FBXW11 in non-small cell lung cancer. *American Journal of Translational Research*.

[14] Xu X., Zheng S. (2020). MiR-887-3p negatively regulates STARD13 and promotes pancreatic cancer progression. *Cancer Management and Research*.

[15] Chen L., Li G., Guo Y., Wan Z., Yu J., Hu W. (2019). Inhibition of miR-9-5p suppresses prostate cancer progress by targeting StarD13. *Cellular & Molecular Biology Letters*.

[16] Nasrallah A., Saykali B., Dimassi S. A., Khoury N., Hanna S., el-Sibai M. I. R. V. A. T. (2014). Effect of StarD13 on colorectal cancer proliferation, motility and invasion. *Oncology Reports*.

[17] Wilbert M. L., Yeo G. W. (2011). Genome-wide approaches in the study of microRNA biology. *Wiley Interdisciplinary Reviews. Systems Biology and Medicine*.

[18] Yang B. F., Lu Y. J., Wang Z. G. (2009). MicroRNAs and apoptosis: implications in the molecular therapy of human disease. *Clinical and Experimental Pharmacology & Physiology*.

The article "miR-182-5p Serves as an Oncogene in Lung Adenocarcinoma through Binding to STARD13" was retracted in 2023. Reasons: signs of a paper mill; suspected computer-generated content; unreliable results or conclusions; lack of ethics approval or compliance.

[19] Cordes K. R., Srivastava D. (2009). MicroRNA regulation of cardiovascular development. *Circulation research*.

[20] Croce C., Calin G. A. (2005). miRNAs, cancer, and stem cell division. *Cell*.

[21] Li Y., Li L. (2019). Prognostic values and prospective pathway signaling of microRNA-182 in ovarian cancer: a study based on gene expression omnibus (GEO) and bioinformatics analysis. *Journal of ovarian research*.

[22] Xue J., Zhou A., Wu Y. (2016). miR-182-5p induced by STAT3 activation promotes glioma tumorigenesis. *Cancer Research*.

[23] Li Y., Chen S., Shan Z. (2017). miR-182-5p improves the viability, mitosis, migration, and invasion ability of human gastric cancer cells by down-regulating RAB27A. *Bioscience reports*.

[24] Yang Q., Tang Y., Tang C. (2019). Diminished LINC00173 expression induced miR-182-5p accumulation promotes cell proliferation, migration and apoptosis inhibition via AGER/NF-*κ*B pathway in non-small-cell lung cancer. *American Journal of Translational Research*.

[25] Ching Y. P., Wong C. M., Chan S. F. (2003). Deleted in liver cancer (DLC) 2 encodes a RhoGAP protein with growth suppressor function and is underexpressed in hepatocellular carcinoma. *The Journal of Biological Chemistry*.

[26] Thorsell A. G., Lee W. H., Persson C. (2011). Comparative structural analysis of lipid binding START domains. *PLoS One*.

[27] Ullmannova V., Popescu N. C. (2006). Expression profile of the tumor suppressor genes DLC-1 and DLC-2 in solid tumors. *International Journal of Oncology*.

[28] Nagaraja G. M., Kandpal R. P. (2004). Chromosome 13q12 encoded Rho GTPase activating protein suppresses growth of breast carcinoma cells, and yeast two-hybrid screen shows its interaction with several proteins. *Biochemical and Biophysical Research Communications*.

[29] Leung T. H., Yam J. W., Chan L. K., Ching Y. P., Ng I. O. (2010). Deleted in liver cancer 2 suppresses cell growth via the regulation of the Raf-1-ERK1/2-p70S6K signalling pathway. *Liver International*.

